# The Effect of Calisthenics on Hypoglycemic of Diabetic Patients

This article has been retracted.

**DOI:** 10.1155/2022/7737626

**Published:** 2022-06-07

**Authors:** Gang Wu, Haili Qu

**Affiliations:** Weifang Engineering Vocational College, China

## Abstract

**Objective:**

To analyze the effect of calisthenics on hypoglycemic in diabetic patients.

**Method:**

From September 2019 to May 2020, 210 patients with type 2 diabetes who were newly diagnosed in our hospital were chosen. They were split into two groups: observation (*n* = 105) and control (*n* = 105). Only drug therapy and diet management were given to the control group, whereas the observation group was given calisthenics treatment in addition to regular diet control and medicine. The outcomes of the two groups of patient's blood glucose levels, BMI, quality of life, and blood lipid index were compared in this study.

**Results:**

Before treatment, there was no significant difference in FPG, 2hPG, and HbA1c levels between the two groups (*P* > 0.05). Compared with before treatment, FPG, 2hPG, and HbA1c were significantly reduced in both groups (*P* < 0.05). In addition, FPG, 2hPG, and HbA1c in the observation group were significantly lower than those in the control group (*P* < 0.05). There was no significant difference in BMI between the two groups before treatment (*P* > 0.05). After treatment, the BMI of the two groups was significantly reduced (*P* < 0.05), and the BMI of the observation group was significantly lower than that of the control group (*P* < 0.05). A comparison of the two groups' SF-36 scale scores before intervention revealed no statistically significant difference (*P* > 0.05). The observation group's SF-36 scores were substantially higher than the control group's after intervention (*P* < 0.05). After treatment, the TC and HDL-c levels in the observation group were not significantly different from those in the control group (*P* > 0.05). Compared with the control group, TG and LDL-C levels were significantly decreased, with statistically significant differences (*P* < 0.05).

**Conclusion:**

Based on routine nursing intervention, using calisthenics to treat blood sugar has a significant effect, it not only made the patient's self-care ability significantly improved, which was worthy of active promotion in clinical practice.

## 1. Introduction

In China, type 2 diabetes mellitus (T2DM) is one of the most common chronic noncommunicable diseases, with a high incidence, various complications, and a high mortality rate [1].Chronic complications of diabetes are the main causes of disability and death of diabetes, including cerebrovascular, cardiovascular and lower limb vascular diseases in macrovascular complications, and kidney and fundus diseases in microvascular complications. Neuropathy includes sensory nerves responsible for senses; motor nerves controlling physical activities; and autonomic neuropathy managing visceral, vascular, and endocrine functions [2, 3]. The key to delaying the advancement of the disease and limiting consequences is to keep blood glucose levels under control. Abnormal glucose tolerance is a type of diabetes that develops early in the course of the disease, when the patient has no visible clinical signs. However, it frequently implies a problem with glucose and lipid metabolism in the body, which can quickly progress to type 2 diabetes [4, 5]. Type 2 diabetes not only plays an important role in postponing or avoiding complications of diabetes but also can reduce the damage to the cardiovascular system and effectively reduce blood glucose and glycosylated hemoglobin. It makes the blood sugar get better control and reduces the dosage of hypoglycemic drugs [6]. Unreasonable exercise, lack of supervision, lack of indications, too intense, for an extended period of time, or fasting, on the other hand, will not only fail to reach the therapeutic goal, but may also result in hypoglycemia [7]. Therefore, it is of great significance to carry out nursing intervention for exercise therapy for diabetic patients. Relevant studies have found that abnormal glucose tolerance is reversible, and moderate aerobic exercise can play a positive role in controlling blood glucose levels, improving quality of life, reducing and delaying diabetes, and caring for the occurrence of cerebrovascular diseases [8] [9].On the basis of hypoglycemic drug therapy, combined with aerobic exercise intervention, patients with type 2 diabetes can effectively improve the control rate of clinical observation indicators [10, 11]. Calisthenics is one of the three basic diabetes therapies, and it relates to diabetic patients' long-term scientific and regular exercise. It has been proven that exercise has a better hypoglycemic effect [12].Aerobics training can improve the immune function and condition of patients with type II diabetes by affecting hemoglobin A1c and T cells [13].The calisthenics of exercise therapy involves many specific links, such as exercise types, intensity, rhythm, and the best time for exercise [9].This study discussed the hypoglycemic effect of Aerobics on diabetes patients through the changes of four indicators (blood glucose; BMI; quality of life; and lipid profile) and achieved satisfactory results. Diabetes patients can alleviate the harm of diabetes through aerobics, and medical staff can also promote aerobics as one of the important rehabilitation methods for diabetes patients. The rest of the paper is organized as follows: Section 2 gives material and methods, Section 3 gives results, there is discussion in Section 4, and the conclusion is given in Section 5.

## 2. Material and Methods

In this section, we will discuss general information, methods, observational index, and statistical methods in detail.

### 2.1. General Information

We selected 210 patients with type II diabetes newly diagnosed in our hospital from September 2019 to may 2020. A simple randomization method was used to randomly allocate 105 cases in each group. In the control group, there were 49 males and 56 females; they were 43 to 72 years old, with an average of 55.43 ± 12.51 years old. The course of the disease was 1 to 5 years, with an average of 3.34 ± 1.49 years. There were 55 cases of hyperlipidemia, 23 cases of fatty liver, and 27 cases of hyperuricemia. In the observation group, there were 51 males and 54 females; they were 42-71 years old, with an average of 54.64 ± 13.31 years old. The course of illness was 1 to 5 years, with an average of 3.30 ± 1.34 years. There were 52 cases of hyperlipidemia, 24 cases of fatty liver, and 29 cases of hyperuricemia. There was no statistically significant difference in general information between the two groups of patients (*P* > 0.05) and approved by the hospital ethics committee. General information is shown in Table 1.

Inclusion criteria are as follows: meeting the diagnostic criteria published in the 2013 China T2DM Prevention and Control Guidelines belong to the stagnant type of phlegm and dampness in the “Diagnosis and TCM Staging and Efficacy Evaluation Standards for Diabetes” [14]; agree to the treatment plan; BMI>25 kg/m2; age 20~70 years old; there were no important diseases such as heartlessness, liver, and kidney; good medication compliance; and did not participate in other clinical trials within 3 months before enrollment.

Exclusion criteria are as follows: allergic constitution or allergic to multiple drugs; pregnant and lactating women; in recent 3 months, the patient had a history of infection and trauma; malignant hypertension, myocardial infarction, severe arrhythmia, acute gout; having severe mental disorders; failing to take medicine as prescribed or having incomplete medical records; and some factors cause acute blood glucose elevation.

### 2.2. Methods

Only drug therapy and diet management were given to the control group, whereas the observation group was given calisthenics treatment in addition to regular diet control and medicine. Calisthenics was divided into three sections: warm-up exercise (5 ~10min), step exercise (15~20 min), and relaxation and recovery exercise (5~10 min). Exercise time was 1~2 h after meals, and each exercise time was 20~30 min, 1~2 times a day, guided by the nurse. The patient sweating after exercise, mild shortness of breath, palpitation, heart beat no more than 120 times / minute, recovered after 20 minutes of rest, and his spirit, sleep and appetite were not affected.

### 2.3. Observational Index

The results of blood glucose, BMI, quality of life, and lipid profile were evaluated in both groups.

#### 2.3.1. Blood Glucose Levels

Before and after therapy, patients' fasting blood was obtained in the early morning (2 h PG was collected 2 h after meal). The heparin anticoagulant tube was filled with 8 mL of peripheral venous blood. The serum was centrifuged for 15 minutes at 3000 r/min after standing for 1 hour. The upper serum was isolated and utilized to measure FPG, 2 h PG, and Hb A1c, among other blood glucose indicators.

#### 2.3.2. BMI

The Body Mass Index (BMI) = body mass index (kg)/height (m)2 was measured at the same time and place before and after treatment.

#### 2.3.3. Quality of Life

Before and after the intervention, we quantitatively evaluated the quality of life of the two groups, including physiological characteristics, physiological function, physical pain, vitality, social function, emotional function, mental health and overall health, and scored them with the simple quality of life scale (SF -36) in two groups. There are a total of eight aspects, each with a score ranging from 0 to 100 points; the greater the score, the higher the quality of life level [15].

#### 2.3.4. Lipid Profile

Select the key indicators of lipid profile: Compare TC (total cholesterol), TG (triglyceride), HDL-C (high density lipoprotein cholesterol), and LDL-C (low density lipoprotein cholesterol), and observe the four indicators of observation group and control group.

### 2.4. Statistical Methods

SPSS 17.0 software was used for statistical analysis, and t-test analysis was used for measurement indicators. *P* < 0.05 was statistically significant.

## 3. Results

In this section, we will discuss the result of blood glucose levels, the result of BMI, the result of the quality of life, and the result of serum lipid parameters in detail.

### 3.1. Result of Blood Glucose Levels

Before treatment, there was no significant difference in FPG, 2hPG, and HbA1c levels between the two groups (*P* > 0.05). Compared with before treatment, FPG, 2hPG, and HbA1c were significantly reduced in both groups (*P* < 0.05). In addition, FPG, 2hPG, and HbA1c in the observation group were significantly lower than those in the control group (*P* < 0.05). The result of blood glucose levels is shown in Table 2.

### 3.2. Result of BMI

There was no significant difference in BMI between the two groups before treatment (*P* > 0.05). After treatment, the BMI of the two groups was significantly reduced (*P* < 0.05), and the BMI of the observation group was significantly lower than that of the control group (*P* < 0.05). The result of BMI is shown in Table 3.

### 3.3. Result of Quality of Life

A comparison of scores of the SF-36 scale before intervention between the two groups showed no statistically significant difference (*P* > 0.05). After the intervention, SF-36 scores in the observation group were significantly higher than those in the control group (*P* < 0.05). The result of the quality of life is shown in Table 4.

### 3.4. Result of Serum Lipid Parameter

After treatment, the TC and HDL-c levels in the observation group were not significantly different from those in the control group (*P* > 0.05). Compared with the control group, TG and LDL-C levels were significantly decreased, with statistically significant differences (*P* < 0.05). The result of the serum lipid parameter is shown in Table 5.

## 4. Discussion

Diabetes is a chronic illness that requires prompt, long-term, and thorough care. Regular moderate-intensity aerobic exercise, in addition to diet control, medication, and psychological treatment, is an essential basic therapy in the treatment of type 2 diabetes [16]. Low and medium intensity aerobic exercise combined with vitamin D supplementation can reduce the level of glycosylated hemoglobin in patients with type 2 diabetes, reduce the weight and BMI of patients with type 2 diabetes, and enhance the static balance of patients [17, 18]. It can increase the number of pancreatic receptors on peripheral tissue cells and improve the sensitivity of the receptor [19]. Calisthenics is an important part of the full treatment of type 2 diabetes; however, patients often have higher compliance with diet control and pharmacological therapy than with exercise therapy during the clinical treatment process. The venue is in the sunshine room, or by playing CDS; each patient learns to exercise along with the TV screen and has a sense of rhythm, which can mobilize the enthusiasm of patients to participate [20, 21].Aerobics can make diabetes patients' weight, chest circumference, waist circumference decrease, systolic blood pressure decrease, diastolic blood pressure increase, and blood glucose and triglyceride decrease significantly [22, 23].Reasonable adjustment of diet structure, good blood glucose monitoring, and moderate aerobic exercise can make skeletal muscle get sufficient oxygen supply. Free fatty acids in the body can be completely oxidized and decomposed for energy, which is conducive to weight loss. It can not only significantly improve the quality of life of patients with glucose tolerance but also play a positive role in the control of blood glucose [24, 25]. Calisthenics is a kind of aerobic exercise designed according to the theory of traditional Chinese medicine [26]. The whole exercise process is slow and gentle, which can carry out endurance training and aerobic exercise without causing too much burden to the body [27]. As a result, for individuals with type 2 diabetes, frequent aerobic exercise of suitable intensity and gradual rhythm, with a heartbeat that is not too fast and gentle breathing after exercise, is an essential treatment [28].

Research in this study showed that before treatment, there was no significant difference in FPG, 2hPG, and HbA1c levels between the two groups (*P* > 0.05). Compared with before treatment, FPG, 2hPG, and HbA1c were significantly reduced in both groups (*P* < 0.05). In addition, FPG, 2hPG, and HbA1c in the observation group were significantly lower than those in the control group (*P* < 0.05). There was no significant difference in BMI between the two groups before treatment (*P* > 0.05). After treatment, the BMI of the two groups was significantly reduced (*P* < 0.05), and the BMI of the observation group was significantly lower than that of the control group (*P* < 0.05). A comparison of scores of the SF-36 scale before intervention between the two groups showed no statistically significant difference (*P* > 0.05). After the intervention, SF-36 scores in the observation group were significantly higher than those in the control group (*P* < 0.05). After treatment, the TC and HDL-c levels in the observation group were not significantly different from those in the control group (*P* > 0.05). Compared with the control group, TG and LDL-C levels were significantly decreased, with statistically significant differences (*P* < 0.05).

## 5. Conclusion

The purpose of this study was to see how calisthenics affected diabetic patients' hypoglycemia. There was no statistically significant difference in the SF-36 scale scores between the two groups before intervention. The observation group's SF-36 ratings were significantly higher than the control group's after the intervention. The observation group's TC and HDL-c values after therapy were not substantially different from the control group. TG and LDL-C values were much lower in the experimental group than in the control group, with statistically significant differences. To summarize, employing calisthenics to treat hypoglycemia has a considerable effect based on routine nursing intervention, which not only considerably improves patients' self-care ability in life, but also can reduce the blood sugar of patients, have obvious effects on weight and blood lipid, and improve the quality of life of patients, and worthy of active promotion in clinical practice.

## Figures and Tables

**Table 1:** General Information.

Groups	Observation group	Control group
Gender (M/F)	51/54	49/56
Age	54.64 ± 13.31	55.43 ± 12.51
BMI	26.71 ± 7.06	25.63 ± 9.01
Weight	75.52 ± 29.31	72.39 ± 22.64
Fasting blood glucose	9.56 ± 2.12	8.35 ± 3.14
2 h blood glucose after meal	15.13 ± 5.66	15.31 ± 6.71
HbA1c	8.17 ± 2.06	8.31 ± 2.52
Triacylglycerol	2.05 ± 2.63	2.23 ± 2.87
Cholesterol	4.88 ± 1.53	4.74 ± 3.35
HDL-C	1.17 ± 4.18	1.04 ± 0.67
LDL-C	3.04 ± 2.02	3.05 ± 2.80

**Table 2:** Result of blood glucose levels.

Groups	Observation group	Control group	
FPG (mmol/L)			
Before	8.25 ± 0.78	8.16 ± 1.01
After	5.32 ± 0.56	6.34 ± 0.61
2hPG (mmol/L)		
Before	11.43 ± 1.45	11.18 ± 1.36
After	7.15 ± 1.26	9.01 ± 1.34
HbA1c (%)		
Before	8.30 ± 0.47	8.17 ± 0.53
After	6.32 ± 0.40	7.10 ± 0.51

**Table 3:** Result of BMI.

Groups	BMI (kg/m^2^)	
	Before	After
Observation group	28.64 ± 2.32	24.54 ± 2.03
Control group	28.04 ± 2.50	26.71 ± 2.06

**Table 4:** Result of quality of life.

Groups	Observation group	Control group
Physiological feature		
Before	60.35 ± 10.15	60.21 ± 10.23
After	74.20 ± 13.02	68.17 ± 12.32
Physiological function		
Before	59.20 ± 11.02	59.44 ± 11.02
After	71.11 ± 12.45	65.12 ± 11.02
Physical pain		
Before	67.02 ± 13.23	67.05 ± 13.10
After	79.37 ± 13.35	73.33 ± 12.24
Vitality		
Before	60.02 ± 10.44	60.08 ± 10.37
After	73.11 ± 12.16	67.46 ± 11.13
Social function		
Before	64.26 ± 12.05	64.42 ± 12.01
After	77.24 ± 13.28	71.20 ± 12.18
Emotional function		
Before	59.33 ± 10.01	60.02 ± 10.12
After	76.80 ± 13.02	69.51 ± 12.01
Mental health		
Before	63.21 ± 11.63	63.37 ± 11.56
After	77.18 ± 13.07	70.37 ± 12.36
Overall health		
Before	62.38 ± 12.81	62.02 ± 12.77
After	74.45 ± 12.37	68.22 ± 10.44

**Table 5:** Result of serum lipid parameter.

Groups	Observation group	Control group
TC		
Before	7.23 ± 2.01	7.30 ± 1.95
After	6.01 ± 1.12	6.02 ± 1.10
TG		
Before	4.12 ± 0.20	3.27 ± 0.61
After	2.05 ± 0.32	1.37 ± 0.24
HDL-C		
Before	2.08 ± 0.31	2.14 ± 0.60
After	1.01 ± 0.22	1.02 ± 0.20
LDL-C		
Before	5.68 ± 1.25	6.20 ± 1.71
After	4.40 ± 1.07	3.10 ± 1.05

## Data Availability

The data used to support the findings of this study are included within the article.
